The article "Teaching Analysis for Visual Communication Design with the Perspective of Digital Technology" was published in 2022. Journal: Comput Math Methods Med.

# Teaching Analysis for Visual Communication Design with the Perspective of Digital Technology

**DOI:** 10.1155/2022/2411811

**Published:** 2022-07-19

**Authors:** Qian Sun, Yingjie Zhu

**Affiliations:** Tangshan Normal University, Tangshan 063000, China

## Abstract

The turn of contemporary visual culture has led to the expansion of the connotation and scope of visual communication design (VCD) education, the generation of new artistic concepts and forms, and the great changes in the subject education system. VCD instruction now has an enhanced teaching environment and operational platform because of the rapid advancement of digital technology. Digital technology is expected to break through traditional learning methods in the future and will be more widely integrated into VCD courses. A topic that must be addressed and explored in the reform and growth of VCD education is how to build a fairer and more inclusive college art education subject system. Therefore, it is particularly important to design a complete VCD teaching evaluation system. In this paper, artificial intelligence technology is applied to the teaching quality evaluation (TQE) system, and a scientific and reliable TQE model is obtained. The main works of this paper are as follows: (1) analyze the background and significance of TQE research, and systematically expound the domestic and foreign research status of TQE, genetic algorithm, and neural network. (2) Using an adaptive mutation evolutionary method, this research builds a TQE system for the VCD course and produces a BPNN model. The adaptive mutation genetic algorithm's convergence speed is considerably faster than the regular genetic algorithms, the optimized neural network's performance is also superior, and the model has a faster convergence time and better prediction accuracy.

## 1. Introduction

With the continuous development of human science and culture, the fields involved in various disciplines continue to expand, and no discipline can exist and develop alone [1]. Influenced by today's diversified social forms, there is a closer connection between the design profession and social needs, especially the market economy society has brought new challenges to us when the VCD education has become diversified [2]. Today's society has entered the era of visual culture, which announces the decline of the centrality of language and print culture, and more importantly, a fundamental change in the way the public grasps the world: change from relying on personal experience and language to relying on vision, images, etc. When people communicate more visually, text-based models may not be able to adequately account for visual experience or visual literacy. Therefore, in the era of visual culture, the course teaching of VCD has more important meaning. We can no longer understand design as a narrow concept, and VCD has gradually surpassed its original scope and moved to a wider and wider field [3]. Diversified visual concepts also imply that new VCD will break the boundaries of traditional design categories and make art design a carrier that can integrate multiple disciplines. Emerging digital technology has ushered in historic shifts in design production and manner. Designers can use digital technology to freely manipulate varied visual data and even generate characters that are not there in the computer, allowing them to change flat objects in their hands into three-dimensional shapes. And perform actions in the three-dimensional interface to make the design more lifelike [4, 5].

The article "Teaching Analysis for Visual Communication Design with the Perspective of Digital Technology" was published in 2022. Journal: Comput Math Methods Med.

The digital revolution has revolutionized VCD from editing, typography, graphic processing, and illustration creation. Digital technology has revolutionized education with its advantages of rapidity, multidimensionality, and convenient storage, broadening the scope of school education and the way students receive knowledge. Students majoring in VCD need to acquire a large number of advanced design concepts and popular ideas in the process of learning. In the past, students could only go to the library or bookstore to buy printed materials. When these materials are obtained, they may not be the latest information. Now, students themselves can access information from schools around the world by searching the database or through the Internet. The teaching environment has also undergone unprecedented changes. Students and teachers can establish a simulated teaching environment through digital technology, so that students in different regions can see the teaching content through the interaction provided in the simulated environment, so that in a short time gain knowledge. Information technology has changed the process and relationship of the interaction of system elements. High and new technologies have also brought about major changes in the responsibilities of teachers. It will no longer be based on dissemination of knowledge, but will focus on cultivating students to master the methods of information processing and the ability to analyze and solve problems [6–8]. Therefore, it has also become a necessary topic in this field to conduct a reasonable TQE in the teaching of VCD. In this context, this paper designs a teaching evaluation index system that conforms to the characteristics of the VCD course and introduces AI technology into teaching. TQE in the field of teaching, promoting the change of teaching evaluation methods and providing a basis for scientific and quantitative evaluation of VCD teaching quality, has great theoretical value and practical value.

The article "Teaching Analysis for Visual Communication Design with the Perspective of Digital Technology" was published in 2022. Journal: Comput Math Methods Med.

The following is the paper's organisation paragraph: Section 2 discusses the associated work. The suggested work's approaches are examined in Section 3. The trials and results are discussed in Section 4. Finally, the research job is completed in Section 5.

## 2. Related Work

Vision and its applications are studied in VCD, which is also a major aspect of modern art design. The term “visual communication design” refers to a print art style that emerged in the middle of the nineteenth century in Europe and the United States as a continuation of the plane. During the World Design Conference in Tokyo, Japan in the 1960s, attendees discovered that vision and image had become autonomous techniques of communication in the media, and that they were becoming increasingly important. Graphic design, art design, stereoscopic picture design, and video design are all included in this scope. In today's fast-changing information society, the impact of various media is expanding, and the content of design performances can no longer include some new information communication channels [9]. These media are becoming increasingly important. As a result, VCD was born. As a design medium, the visual media of VCD expresses the time and the rich connotations of design in a way that conveys its message. A new area of design is being formed that is linked to and collaborative with other visual media as science and technology, as well as the creation and use of product materials, continue to evolve. Visual communication is the use of vision as a medium to convey information, that is to say, as long as it is a design field associated with visual media, it should belong to the category of VCD [10]. In this sense, VCD is not only flat but also spatial and dynamic, which contains the trend of future design. Neither type of design can look at it from a graphic design perspective alone. VCD education moves from the classroom to the point-to-point learning between designers. As a new discipline, VCD has great particularity. Teaching and learning are not only done in a typical classroom setting; they are also done via the use of current educational tools, such as videoconferencing and online learning resources. The age of design necessitates that education in design follow suit [11]. Therefore, the TQE of VCD course is also extremely important. Many educators have spent a long time trying to figure out how to create and develop an objective and scientific TQE system. In this regard, countries such as the United Kingdom and the United States got a head start and built on their successes, advancing important ideas and approaches such as multiple intelligences theory, constructivism theory, and the Taylor evaluation model [12]. TQE has been classified into five stages since its inception in the second half of the nineteenth century, according to the features of each period: examination, test, description, reflection, and construction [13]. The initial teaching evaluation exists in the form of examinations, and the results are largely influenced by teachers' subjective judgments.

The article "Teaching Analysis for Visual Communication Design with the Perspective of Digital Technology" was published in 2022. Journal: Comput Math Methods Med.

Since the birth of the concept of teaching evaluation, the development and needs of education have inspired many educators to continuously explore and improve and have also achieved some experience and results. For example, the book “Introduction to Psychological and Social Measurement” published by a famous American educator, the author expresses his thoughts and understanding of educational standardization and puts forward the relevant theoretical basis. This book marks the maturity of educational measurement [14]. Measurement methods such as “Bina-Simon Scale” and TCBE measurement compilation method were born and published one after another, which marked the further maturity of educational measurement [15]. Many scholars in the field of education have successively proposed various TQE models. Reference [16] uses the fuzzy algorithm to establish a quality evaluation system to improve the school's TQE. It can also conduct self-evaluation in stages according to the actual situation of students. Reference [17] used the analytic hierarchy process to quantitatively evaluate the teaching quality of colleges and universities and formed a corresponding evaluation system. Reference [18] constructed a set of teaching quality monitoring system based on the concept of “people-oriented, three-dimensional integration.” “People-oriented” in the system mainly refers to teachers and students-oriented, while “three-dimensional” refers to schools, secondary colleges, teachers, etc. In order to improve the TQE, reference [19] uses the mathematical fuzzy analytic hierarchy process and adds a range of assessment methodologies. Reference [20] created a blended TQE model based on the implementation process of the blended teaching paradigm. Useful outcomes have been obtained in practical applications. Because of the varying understanding and attention on teaching quality, there are some differences in the content and methods of assessment in various schools and institutions [21]. TQE approaches include expert evaluation, fuzzy comprehensive evaluation, neural network model method, and others, according to the available literature. These techniques have their unique evaluation characteristics [22]. Reference [23] uses BPNN and related theories to formulate the evaluation index system, constructs an effective computer graphics TQE model, and uses this model to evaluate the actual teaching situation of related courses. Reference [24] proposed an optimized BP algorithm, and the results after applying it to actual training show that the evaluation model established by this algorithm has fast convergence speed and high accuracy and has broad application prospects in teaching evaluation problems in higher education. Reference [25] combined AHP and neural network, combined the advantages of the two, added a screening process in the evaluation, and finally obtained the AHP-BPNN evaluation model. The PSO algorithm is combined with the neural network in reference [26], and the PSO algorithm is used to optimize the neural network and identify the globally optimal network parameters, resulting in a full TQE evaluation model.

The article "Teaching Analysis for Visual Communication Design with the Perspective of Digital Technology" was published in 2022. Journal: Comput Math Methods Med.

## 3. Method

In this section, we define the principle of the BP neural network, adaptive mutation genetic algorithm steps, improved BP network model, and visual communication design teaching quality evaluation index system in detail.

### 3.1. The Principle of BP Neural Network

The forward transmission of information and the backward propagation of errors make up the BPNN. As soon as data is entered into the network, it begins to spread outward across the input layer of the network. To check whether this mistake fulfills the output result's criteria, the data is sent to the output layer after being processed and computed at each subsequent layer and propagated backwards through several layers of processing. If the fault is significant, it is sent back to the network, and the connection weight threshold between each unit is set at the same time. The neural network continues to propagate through these two phases once the output and conditions are met. Layers 1, 2, and 3 comprise the input, hidden, and output portions of a BPNN, as shown in Figure 1.

When using the BP method of learning, a forward propagation and a back propagation procedure are used in tandem. In a nutshell, the algorithm works like this:

1. The input vector is propagated in the reverse direction. To create the output vector, the input vector is first transported to the hidden layer through the input layer and then to the output layer. The weights of neural networks are not changed while they are sent. If the desired output is not met at the output layer, error back-propagation happens
2. Error propagation is backwards. There are two layers of transmission: one between output and hidden layers, and one between hidden layers and input layers. During the error back-propagation stage, the neural network's weights are continually modified and rectified by the error feedback mechanism, and repeated iterations bring the network output to the intended output

The main idea of the BP learning algorithm is for *q* training samples, *P*_1_, *P*_2_, ⋯, *P*_*q*_, the corresponding output samples are *T*_1_, *T*_2_, ⋯, *T*_*q*_. The goal of learning is to correct the weights by making the error between the target vector *T*_1_, *T*_2_, ⋯, *T*_*q*_ and the actual output *A*_1_, *A*_2_, ⋯, *A*_*q*_, so that the actual output *A*_*i*_(*i* = 1, 2, ⋯, *q*) approaches the expected value *T*_*q*_, and the sum of squares of the network errors is minimized. The calculation steps of the BP algorithm are as follows.

1. Forward transmission of information; the output of the *i*th neuron in the hidden layer, as shown in the following formula

(1) $$\begin{array}{c} y_{h_{i}}=fh\left(wh_{ij}p_{j}+ah_{i}\right),i=1,2,\cdots ,m. \end{array}$$

The output of the *k*th neuron in the output layer is shown in the following formula

(2) $$\begin{array}{c} y_{O_{k}}=fO\left(\overset{n}{\underset{i=1}{\sum }}wO_{ki}y_{h_{i}}+aO_{k}\right),k=1,2,\cdots ,n. \end{array}$$

Define the error function, as shown in the following formula

(3) $$\begin{array}{c} E=\frac{1}{2}\overset{n}{\underset{k=1}{\sum }}{\left(t_{k}-y_{O_{k}}\right)}^{2}. \end{array}$$

(2) Use the gradient descent method to calculate the weight change and the back-propagation of the error. The weight change of the output layer is the weight from the *i*th input to the *k*th output, as shown in the following formula

(4) $$\begin{array}{c} ∆wO_{ki}=-\mu \frac{\partial E}{\partial wO_{ki}}=-\mu \frac{\partial E}{\partial y_{O_{k}}}\times \frac{\partial y_{O_{k}}}{\partial wO_{ki}}=\mu \delta_{ki}y_{h_{i}}. \end{array}$$

The hidden layer weight changes, for the weight from the *j*th input to the *i*th output, as shown in the following formula

(5) $$\begin{array}{c} ∆wh_{ki}=-\mu \frac{\partial E}{\partial wh_{ki}}=-\mu \frac{\partial E}{\partial y_{O_{k}}}\times \frac{\partial y_{O_{k}}}{\partial wh_{ki}}=\mu \delta_{ij}h_{ki}. \end{array}$$

The weights and thresholds of each layer in the network should be changed, and the next training sample should be selected and fed into the input layer until all samples in the training set are learnt. If the result's error range falls within a certain range, the training may be repeated as many times as necessary to bring it into compliance. Training has been completed, so save the neural network for future use and stop.

The article "Teaching Analysis for Visual Communication Design with the Perspective of Digital Technology" was published in 2022. Journal: Comput Math Methods Med.

### 3.2. Adaptive Mutation Genetic Algorithm Steps

1. Genetic algorithms do not directly look for possible answers in the process of addressing actual issues. It is instead encoded first, and encoding strategy has a significant impact on the genetic algorithm's ability to find the best global solution. Binary, sequence, real number, tree, out-of-order, and huge character set encoding are some of the most common genetic algorithm encoding techniques
2. There are a number of ways to determine the number of first solutions. For a global optimum solution to be discovered, a large beginning population is necessary. However, a larger starting population will need more fitness function computations, reducing the efficiency of the solution. As a result, there can be no extremes in terms of the size of the beginning population. Schaffer recommended a population size of between [20, 100]. A series of trials have shown that the least error, 0.2135, and the quickest convergence time occur when the starting population is 20. The starting population of 20 is used in this work
3. *Calculation of Fitness*. With an eye on improving fitness function, the genetic algorithm aims to find network weights and thresholds that minimize the network's total squared errors throughout all evolutionary generations. To that end, it adjusts network weights and thresholds in order to maximize fitness function. The learning error is shown in formula (6), and the fitness function is shown in formula (7).

(6) $$\begin{array}{c} E=\frac{\sum_{k=1}^{n}\sum_{j=1}^{m}\left(y_{j}^{k}-O_{j}^{k}\right)}{2}, \end{array}$$

(7) $$\begin{array}{c} \text{Fit}=\frac{1}{E}, \end{array}$$

where *E* is the learning error, *n* is the number of training samples, *m* is the number of output nodes, and *y*_*j*_^*k*^ − *O*_*j*_^*k*^ is the error of the kth sample relative to the *j*th output node.

(4) *Genetic Operation*. Proportional selection, or replication, is the strategy used in this study. For each generation of people, the weight and threshold of the BP neural network are utilized to calculate the fitness value. Then, the entire fitness value is determined. An individual is more likely to be selected for further evaluation if their fitness values make up a larger proportion of their overall score. The formula for calculating the likelihood of selection is presented in the following equation below.

(8) $$\begin{array}{c} C\left(u_{j}\right)=\frac{f\left(u_{j}\right)}{\sum_{j=1}^{P}f\left(u_{j}\right)}, \end{array}$$

where *u*_*j*_ represents an individual in the group, *C*(*u*_*j*_) is the probability that *u*_*j*_ is selected, *f*(*u*_*j*_) is the fitness value of individual *u*_*j*_, and *P* is the population size.

In order to establish if a selected person may be passed down to future generations, it is required to compute the likelihood that the selected individual will be chosen. The calculation formula is shown in the following formula.

(9) $$\begin{array}{c} p\left(u_{k}\right)=\overset{k}{\underset{j=1}{\sum }}C\left(u_{j}\right), \end{array}$$

where *p*(*u*_*k*_) is the cumulative probability of individual *u*_*k*_, then a new population of the next generation is obtained through genetic manipulation, the fitness value is judged, and the above steps are repeated until the population is stable.

The article "Teaching Analysis for Visual Communication Design with the Perspective of Digital Technology" was published in 2022. Journal: Comput Math Methods Med.

It is the crossover operation in genetics that enables the creation of new people by exchanging a few genes. New gene structures are introduced more quickly in a population where the crossover probability is high, whereas the loss rate of previously discovered, highly effective gene structures are comparatively high in a population where the crossover probability is low. [0.6, 1.0] is the typical crossover probability range.

During the mutation process, some of the population's genes get mutated at a predefined pace. The adaptive mutation probability mutation operation is used in the model. There will be some undesirable shapes, but in general, the genetic algorithm's population will become more diverse as a result of the process of mutation, which retains some good mutations. As soon as possible, it leaves the local optimal situation, seeks for the optimal solution at the global level, and steers clear of any premature phenomena.

### 3.3. Improved BP Network Model

#### 3.3.1. AGA-BP Model

The BPNN relies heavily on its starting weights and thresholds, which are provided at random. Many researchers use new optimization strategies to enhance the neural network. Genomic algorithms, for example, are often used to enhance the neural network. As a result, the genetic algorithm may enhance the neural network based on gradient descent, which has a tendency to fall into a local minimum value and a sluggish convergence speed, by searching for the best solution in the whole space. The BPNN is improved using a genetic method that uses adaptive mutation. It is called the AGA-BPNN, and it has two parts: the BPNN and the AGA. The BPNN design process may be summarized as follows.

1. Multiple-layer feedforward neural networks only need two hidden layers for learning discontinuous functions. A hidden layer should be put up initially when creating a feedforward neural network with several layers. When the network's hidden layer nodes increase in number without improving performance, training expenses rise. As a consequence, this research attempts to use a hidden layer for the first time. This layer's number of nodes is governed by the input vector's size from the outside. A linear transfer function, *f*(*x*) = *x*, characterizes the input layer's transfer function in general. Trial and error is one method for determining the number of hidden layer nodes. It is possible to undertake experiments to determine the optimal number of hidden layers by increasing the number of hidden layers once a starting value has been determined. The number of hidden layer nodes may be calculated using the trial and error method employed in this study:

(10) $$\begin{array}{c} h=\sqrt{i+j}+b, \end{array}$$

where *h* is the number of hidden layer nodes, *i* is the number of input layer nodes, *j* is the number of output layer nodes, and *b* is a constant between 1 and 10.

(2) Obtain data samples and do data preprocessing to determine the number of samples. To a certain extent, greater numbers of experimental samples lead to more precise reactions, but at a certain point, the precision is fixed within a range and cannot be altered. As the network grows in size, the mapping connection becomes increasingly complicated. The entire number of network connection weights is often 5-10 times more than the total number of training samples
(3) It is possible to choose the weights of the network in two different methods. As a first step, you may either choose a low beginning weight, or you can have both weights start at the same amount
(4) Cycle training's weight loss is greatly influenced by the individual's pace of weight gain. Increasing the value will result in system instability, while decreasing it will result in an increased training time but a guaranteed error range
(5) In order to terminate training, there are two options: one is to control over the error range, and the other is to achieve the maximum number of iterations possible. If one of the two prerequisites is met, the training can be halted. Typically, several networks are trained, and the best one is picked based on the research findings. The final AGA-BP algorithm model is shown in Figure 2

The AGA-BP algorithm model includes the flowchart of the BPNN and the adaptive mutation genetic algorithm. The optimal solution searched by the genetic algorithm is input into the BPNN as the initial weight and threshold of the network. Among them, the data flow of the model is as follows. AGA-BP algorithm model inputs begin with the BPNN portion. A neural network's topology, or the number of layers and neurons inside each layer, may be derived from the data acquired via the questionnaire. To find a solution that satisfies the stopping condition, that is, the optimal weight and threshold, the data information processing part begins with the genetic algorithm part of the adaptive mutation. Coding, fitness calculations, genetic operations, and other processes follow. It can lessen the time it takes to discover the best weights and thresholds to speed up network convergence. A better AGA-BP algorithm model is produced if the learning error of the sample or the number of iterations fulfills the conditions.

The article "Teaching Analysis for Visual Communication Design with the Perspective of Digital Technology" was published in 2022. Journal: Comput Math Methods Med.

#### 3.3.2. EM-AGA-BP Model

The entropy method, improved genetic algorithm, and neural network are combined to establish a TQE model, which is named EM-AGA-BP model. The adaptive mutation probability is adopted in the genetic operation process, which not only improves the speed of neural network convergence but also reduces the complexity of the training process. The model not only exerts the advantages of improved genetic algorithm global search and BPNN in nonlinear mapping but also reduces the influence of nonobjective factors. The main modeling steps of the TQE model are as follows:

1. By analyzing the existing problems of TQE, improving them, and establishing a more perfect and more suitable index system
2. TQE sample data should be gathered, and instructors' instructional qualities should be taken into consideration while selecting assessment indicators
3. BPNN parameters include learning rate, hidden layer number of neurons, maximum number of iterations, minimal error accuracy, transfer function, and training durations, and they need all be determined
4. Iterative training is performed until the algorithm is prompted to stop by using the evaluation model
5. Input the test samples for TQE to test whether the training effect of the EM-AGA-BP algorithm meets the requirements. If the prediction results meet the stopping requirements, go to the next step; otherwise, go back to the previous step and retrain the network, that is, go back to step (3).
6. Input the sample into the TQE model to get the TQE result

### 3.4. Visual Communication Design Teaching Quality Evaluation Index System

Different types of schools and courses have different characteristics and have different advantages and characteristics for the development of students. If the TQE system converges, it will make it difficult for the evaluation results to effectively and truly reflect on the essential level of teaching quality. All types of schools should strictly follow the standards and requirements for personnel training formulated by the national education policy and combine the actual situation of schools and courses to clarify their own school-running advantages and shortcomings and propose appropriate and reasonable scientific school-running goals and requirements. The consistency and similarity of the curriculum are transformed into the characteristics and differences of the curriculum. Schools need to update their own teaching models and methods in a timely manner according to the needs of the society. Individual growth, commonality, uniqueness, the common law of teaching, and the teaching characteristics of various types and degrees of school instructors should all be considered while building a TQE system. TQE standards are important at this time because they can assist prevent waste of educational resources and make efficient use of those that are available through a system that is diverse, reasonable, and unique. Survey results were used to identify and prioritize issues in current TQE systems and then used AI and other nonlinear problem-solving methods to design a suitable TQE index system. It was determined that the previous TQE system was flawed, and a TQE model was developed based on an investigation into literature and the TQE index systems of other schools and institutions, which led to the improvement of the system.  Table 1 illustrates the new TQE index scheme. Five levels of quality are assigned to the TQE findings as a consequence of the neural network's work: excellent, good, medium, and pass/fail.

The article "Teaching Analysis for Visual Communication Design with the Perspective of Digital Technology" was published in 2022. Journal: Comput Math Methods Med.

## 4. Experiment and Analysis

In the experiment and analysis section, we discuss the data collection and preprocessing, determination of parameters, and testing the neural network model in depth.

### 4.1. Data Collection and Preprocessing

It is customary to conduct a questionnaire survey in order to gather data. An index system is developed, a questionnaire is created, and a return questionnaire is sent in this research, which incorporates relevant theory and practice of instructors' TQE. Multiple-choice and open-ended items are both included in the questionnaire we developed for this study. To take the TQE approach as an example, the first section of the course consists of multiple-choice questions. The TQE index system's five first-level indicators and sixteen second-level indicators are used to construct multiple-choice questions, with the most appropriate one chosen from various assessment levels for each index. It is required to provide numerical values to each choice after picking the most suited one, since this paper's questionnaire is quantitative in nature. The second section of the question is completely open-ended. When it comes to calculating the overall questionnaire score, this section is not included. Students in a school's VCD program are the focus of a questionnaire survey. There were approximately 1,300 questionnaires distributed, 1,350 of which were retrieved, and 1,200 valid questionnaires were evaluated, totaling 1,200 pieces of valid data. [0, 100] was standardized to between [0, 1] according to the results of the aforementioned questionnaire. To maintain as much of the data's original meaning as possible, this study uses the maximum and minimum procedures, which are two of the most frequent normalizing techniques. The calculation of this method is shown in the following formula

(11) $$\begin{array}{c} X=\frac{S-S_{\min}}{S_{\max}-S_{\min}}, \end{array}$$

where *X* is the normalized score, that is, the input value of the entropy method, *S*_min_ is the minimum teaching quality score, *S*_max_ is the maximum score, and *S* is the unprocessed score.

The article "Teaching Analysis for Visual Communication Design with the Perspective of Digital Technology" was published in 2022. Journal: Comput Math Methods Med.

### 4.2. Determination of Parameters

#### 4.2.1. Determination of Adaptive Genetic Algorithm Parameters

The initial population size in this work is set at 20, 30, and 40 in accordance with the range of the initial population size, and experiments are carried out to acquire the population size training outcomes, in order to get a better initial population size, see it in Figures 3 and 4.

According to Figures 3 and 4, as can be observed, the convergence time is quickest, and the error is least when the starting population size is 20. Therefore, an initial population size of 20 is obtained. Set the crossover probability to 0.65. For the more complex solution space, the real number coding method can be used without decoding. It is thus necessary to utilize this coding strategy in order to code the possible solutions before applying BPNN weights and thresholds. The hidden layer threshold, the hidden layer weight, the hidden layer weight to the output layer, and the output layer threshold make up this system.

#### 4.2.2. Determination of BP Neural Network Parameters

In practice, the most difficult tasks may be solved using a three-layer neural network. The number of layers may be raised in order to enhance the accuracy, but this will make the network more difficult. Increasing the number of neurons in the buried layer may help improve the mistake rate. From the perspective of structure realization, the method of adding hidden layer nodes is simpler than adding more hidden layers, and the training effect is easier to observe and adjust. In order to improve the network's accuracy and efficiency, this study employs the strategy of altering the number of hidden layer nodes. Using the TQE model of the study, the neural network is configured to have one hidden layer, a three-layer neural network.

The number of secondary indicators in the theoretical TQE system is 16; hence, the number of neurons in the input layer is determined to be 16. The number of neurons in the hidden layer may be determined using this method: multiple networks are created with 5 nodes in the hidden layer, and the number of nodes in each network's hidden layer is raised by 1 based on the empirical formula.  Figure 5 shows the experimental outcomes. There are six hidden layers in the BPNN, and as can be seen, this yields the lowest error when there are six nodes buried under the surface. The number of neurons in the output layer is determined by the output target, which is the TQE result.

The article "Teaching Analysis for Visual Communication Design with the Perspective of Digital Technology" was published in 2022. Journal: Comput Math Methods Med.

### 4.3. Testing the Neural Network Model

Since the indicators of the TQE system established in this paper are all positive indicators, the data translation step is omitted, and the entropy approach is used to calculate the weights of the TQE indicators. The transfer function used in this paper's neural network output layer is an S-function, and its output is limited to (0 to 1), so the neural network output range is limited to (0 to 1) as a result (0,1). The range of the initial value of TQE determined by the entropy value method is (0,1), so data standardization is performed again. A total of 1200 groups of data were finally determined to participate in the experiment, of which 1000 groups were used for training the model so that the optimized BPNN structure could be obtained, and the remaining 200 groups of data were used for testing. The data of 16 secondary indicators as the input value of the network test, based on the entropy value technique, are contained in the 1-16 columns of each set of samples. The preliminary evaluation result is the output target of the network. After continuous learning, after obtaining an ideal model, input the score data of the TQE index of the 1001st~1200th group, and the neural network predicts and outputs the TQE results. Part of the experimental results is shown in Figure 6.

The results of the final experiment are shown in Table 2. The BPNN model's average evaluation accuracy for 200 sets of data is 85.37%, the AGA-BPNN model's average evaluation accuracy is 90.76%, and the EM-AGA-BP algorithm's average evaluation accuracy is 97.65%, an increase of 12.28% and 6.89%, respectively. It can be seen that the EM-AGA-BP algorithm has better evaluation results.

## 5. Conclusion

In the digital age, in order to achieve the expected purpose, the VCD course must improve the technological content and inject new connotations and characteristics of the times. The rapid development of digital technology provides an advanced teaching environment and operating platform for VCD teaching. Multimedia technology combines high integration, great interactivity, and a significant volume of data to give rich graphics, images, sounds, and text information. Multimedia technology is expected to fundamentally disrupt traditional learning methods in the future and become more widely integrated into VCD courses. Therefore, while inheriting the past cultural heritage and subject foundation, we must vigorously promote the integration of digital technology and curriculum reform, absorb high-tech achievements, improve teachers' computer-aided teaching level, and extend the curriculum content to the level of intelligence and automation. As a result, developing a comprehensive VCD teaching assessment system is critical. In this study, AI is applied to the TQE system, resulting in a scientific and reliable TQE model. The main works of this paper are as follows: (1) analyze the background and significance of TQE research, and systematically expound the domestic and foreign research status of TQE, genetic algorithm, and neural network. (2) According to the characteristics of the VCD course, this paper builds a TQE system for VCD that is more in line with the characteristics of the digital age. (3) The genetic algorithm and the BPNN model are combined to generate an adaptive mutation method that can be used to improve the initial threshold and weight of the BPNN model. The EM-AGA-BP algorithm is then created. An enhanced convergence time and better neural network performance have been shown by experimental data, which show that the EM-AGA-BP method outperforms classic genetic algorithms, and its convergence time and accuracy are better with the TQE model.

The article "Teaching Analysis for Visual Communication Design with the Perspective of Digital Technology" was published in 2022. Journal: Comput Math Methods Med.

## Figures and Tables

**Figure 1:** BP neural network structure diagram.

**Figure 2:** AGA-BP algorithm model.

**Figure 3:** Comparison of convergence time for different population sizes.

**Figure 4:** Comparison of error for different population sizes.

**Figure 5:** The number of hidden layer nodes and the corresponding error.

**Figure 6:** Experiment results of teaching quality evaluation model.

**Table 1:** Visual communication design teaching quality evaluation index system.

First-level indicator	Secondary indicators	Label
Teacher quality	Educational goals are clear	X1
	Solid professional knowledge	X2
	Excellent teaching level	X3
Teaching attitude	Counseling patiently and actively	X4
	The teaching is conscientious and contagious	X5
	Rigorous attitude and excellence	X6
Teaching content	Concept theory is accurate and novel	X7
	Content-rich, attention-seeking exercise	X8
	Connect with reality and focus on skill training	X9
	Expertise with depth and breadth	X10
Teaching method	Good at inspiring, leading thinking	X11
	Variety of ways, appropriate citations	X12
	Teaching students according to their aptitude	X13
Teaching effect	Good basic knowledge	X14
	Improve self-learning ability and interest in learning	X15
	Improve comprehensive quality and innovation ability	X16

The article "Teaching Analysis for Visual Communication Design with the Perspective of Digital Technology" was published in 2022. Journal: Comput Math Methods Med.

**Table 2:** Average evaluation accuracy of each network model.

Evaluation model	Prediction accuracy
BP neural network	85.37%
AGA-BP algorithm	90.76%
EM-AGA-BP algorithm	97.65%

## Data Availability

The datasets used during the current study are available from the corresponding author on reasonable request.
